The article "Inhibition of Tumor Vasculogenic Mimicry and Prolongation of Host Survival in Highly Aggressive Gallbladder Cancers by Norcantharidin via Blocking the Ephrin Type a Receptor 2/Focal Adhesion Kinase/Paxillin Signaling Pathway" was retracted in 2025. Reasons: plagiarized data; plagiarized images; duplicated images; duplicated data.

# Inhibition of Tumor Vasculogenic Mimicry and Prolongation of Host Survival in Highly Aggressive Gallbladder Cancers by Norcantharidin *via* Blocking the Ephrin Type a Receptor 2/Focal Adhesion Kinase/Paxillin Signaling Pathway

**DOI:** 10.1371/journal.pone.0096982

**Published:** 2014-05-08

**Authors:** Hui Wang, Wei Sun, Wen-Zhong Zhang, Chun-Yan Ge, Jing-Tao Zhang, Zhong-Yan Liu, Yue-Zu Fan

**Affiliations:** 1 Department of Surgery, Tongji Hospital, Tongji University School of Medicine, Tongji University, Shanghai, P.R. China; 2 Department of Surgery, Shanghai Tenth People's Hospital, Tongji University School of Medicine, Tongji University, Shanghai, P.R. China; 3 Department of Surgery, Shanghai Pudong New Area People's Hospital, Shanghai, P.R. China; 4 Department of Oncology, Shanghai Yangpu Geriatric Hospital, Shanghai, P.R. China; Sun Yat-sen University Medical School, China

## Abstract

Vasculogenic mimicry (VM) is a newly-defined tumor microcirculation pattern in highly aggressive malignant tumors. We recently reported tumor growth and VM formation of gallbladder cancers through the contribution of the ephrin type a receptor 2 (EphA2)/focal adhesion kinase (FAK)/Paxillin signaling pathways. In this study, we further investigated the anti-VM activity of norcantharidin (NCTD) as a VM inhibitor for gallbladder cancers and the underlying mechanisms. *In vivo* and *in vitro* experiments to determine the effects of NCTD on tumor growth, host survival, VM formation of GBC-SD nude mouse xenografts, and vasculogenic-like networks, malignant phenotypes i.e., proliferation, apoptosis, invasion and migration of GBC-SD cells. Expression of VM signaling-related markers EphA2, FAK and Paxillin *in vivo* and *in vitro* were examined by immunofluorescence, western blotting and real-time polymerase chain reaction (RT-PCR), respectively. The results showed that after treatment with NCTD, GBC-SD cells were unable to form VM structures when injecting into nude mouse, growth of the xenograft was inhibited and these observations were confirmed by facts that VM formation by three-dimensional (3-D) matrix, proliferation, apoptosis, invasion, migration of GBC-SD cells were affected; and survival time of the xenograft mice was prolonged. Furthermore, expression of EphA2, FAK and Paxillin proteins/mRNAs of the xenografts was downregulated. Thus, we concluded that NCTD has potential anti-VM activity against human gallbladder cancers; one of the underlying mechanisms may be *via* blocking the EphA2/FAK/Paxillin signaling pathway.

## Introduction

Gallbladder cancer (GBC), a lethal aggressive malignant neoplasm, is the most common malignancy of the biliary tract, the 5th or 6th common malignant neoplasm of the digestive tract and the leading cause of cancer-related deaths in Western countries and China [1]–[3]. Despite significant breakthroughs in understanding the pathology and biological behavior of the tumor, survival and prognosis of these patients is still very poor [1], [4], [5]. Especially, highly aggressive gallbladder cancer is a considerable clinical problem not only due to diagnostic delay, dismal results of surgical resection, chemotherapy and radiotherapy for the disease, but also due to the complexity of targeting the elusive metastatic phenotypes [1], [6]–[9].

Research has shown that the plastic notion of some highly aggressive tumor such as melanoma is characterized by the concurrent expression of genes from a variety of different cell types, including stem cells, concomitantly with reduced melanoma associate gene expression [10]. In particular, highly aggressive melanoma cells, in contrast to poorly aggressive ones, display substantial plasticity, exemplified by the formation of tube-like structures termed Vasculogenic mimicry (VM) [11]. These structures are comprised exclusively of tumor cells but not of endothelial cells, and conduct blood cells and fluids. Similarly, we found that the plastic notion of gallbladder cancer is characterized by the concurrent expression of genes from a variety of different cell types, such as highly aggressive GBC-SD cells and poorly aggressive SGC-996 cells. Highly aggressive GBC-SD cells formed VM-like network structures by both 3-D matrices *in vitr*o and nude mouse xenografts *in vivo*, whereas poorly aggressive SGC-996 cells did not form the vasculogenic-like networks under the same conditions, but formed pattern, vasculogenic-like networks when cultured on a matrix preconditioned by the GBC-SD cells [12], [13].

VM, independently of angiogenesis and vasculogenesis, is a novel paravascular tumor blood supply pattern in some highly aggressive malignant tumors formed by tumor cells instead of endothelial cells [11]. VM describes the unique ability of highly aggressive tumor cells to express endothelial cell-associated genes and form extracellular matrix (ECM)-rich, patterned tubular networks when cultured on a 3-D matrix [11]. In histology, VM emerges as multiple, ECM-rich networks surrounding clusters of tumor cells, which can be stained with periodic acid-Schiff (PAS) [11]. VM or a PAS-positive pattern is associated with tumor aggressiveness, poor clinical outcome, and high risk of recurrence in patients with melanoma [11], [14]–[16], gallbladder cancer [17], [18], and other malignances [19]–[22]. Because the formation of VM channels is not an angiogenic event as it does not arise from pre-existing vessels, this angiogenesis-independent fact could explain why antiangiogenic therapies have clinically failed in some tumors, specially highly aggressive tumors e.g. melanoma, despite being macroscopically a highly “vascular” tumor [23]–[25]. Indeed, some antiangiogenic drugs, such as bevacizumab, sorafenib and endostatin, have been ineffective at inhibiting VM [26]–[28].

Since VM is an alternative pathway for tumors to guarantee their blood supply, it is necessary to find potential therapeutic approaches that could target this alternative vascular pathway. Currently, many researchers are seeking to develop new VM inhibitors from cleaved proteins, monoclonal antibodies, synthesized small molecules and natural products [25], [29]–[32]. However, there is no experimental or clinical inhibitor for gallbladder cancer VM. Thus, in view of worse treatment results, poor prognosis and special biological behavior in the patients with gallbladder cancer, it should be considered to develop novel anti-VM therapeutic agents that target VM when in antitumor treatment of highly aggressive tumors, to further develop more effective comprehensive therapies such as combining anti-VM or anti-angiogenic drugs with conventional chemotherapies, or traditional Chinese medicines which have multifunctional antitumor activities.

NCTD is a demethylated form and low-cytotoxic derivative of cantharidin with antitumor properties, and is an active ingredient of the traditional Chinese medicine *Mylabris*, also is synthesized from furan and maleic anhydride *via* the Diels Alder reaction [33]–[35]. It has been reported that NCTD inhibits the growth of a variety of human tumor cells, including HepG2, K562, HL60, A375-S2, HT29 and GBC-SD cells, and is clinically used to treat human cancers, e.g., hepatic, gastric, colorectal and ovarian cancers [33]–[38]. We have reported that NCTD has multiple antitumor activities against gallbladder cancers *in vitro* and *in vivo* [39]–[41]. However the exact mechanism responsible for the NCTD antitumor is not thoroughly elucidated. We recently reported that VM existed in human gallbladder cancers and gallbladder cancers by both 3-D matrix of highly aggressive GBC-SD cells *in vitro* and GBC-SD nude mouse xenografts *in vivo* and correlated with the patient's poor prognosis and that poorly aggressive SGC-996 cells did not form the vasculogenic-like networks when cultured under the same conditions [12], [13], [17], [18]. We identified that VM formation in gallbladder cancers through the activation of a key VM-related signaling pathway—the EphA2/FAK/Paxillin signaling pathway in the 3-D matrix of highly aggressive GBC-SD cells *in vitro* and GBC-SD nude mouse xenografts *in vivo* [42]. In this study, we firstly show evidence that NCTD inhibits tumor VM and prolongs host survival in highly aggressive gallbladder cancers *via* blocking the EphA2/FAK/Paxillin signaling pathway, thus may serve as a potential target inhibitor for VM of highly aggressive gallbladder cancers.

## Results

### NCTD inhibits tumor growth, prolongs host survival and suppresses VM formation of GBC-SD nude mouse xenografts *in vivo*

We previously reported that NCTD has multiple antitumor activities against gallbladder cancers, while tissue inhibitor of matrix metalloproteinase-2 (TIMP-2, a 21-kDa protein and VM inhibitor) has anti-VM activity for these cancers [39]-[42]. Here, we investigated anti-VM activity of NCTD for highly aggressive gallbladder cancer *via* VM formation and tumor assays of GBC-SD nude mouse xenografts and a survival analysis of xenograft mice. In the experiment, GBC-SD xenografts appeared gradually in subcutaneous area of the right-rear axils of nude mice from the 6th day after inoculation, were in all nude mice after 3 weeks. In NCTD group, the xenograft volume was markedly decreased, tumor inhibition was significantly increased as compared to control group (Fig.1A and 1B; all *p*<0.001), and the tumor inhibition was much higher than that of TIMP-2 group (Fig.1B; *p*<0.01). Furthermore, the xenograft mice were all alive at the end of the experiments, with prolonged survival time in NCTD group when compared with control group (Fig.1C; log-rank test, *p* = 0.022).

**Figure 1:** Effects of NCTD on growth of GBC-SD nude mouse xenografts and survival of the xenograft mice *in vivo*. (**A**) Growth inhibition curves (tumor volume, cm^3^) of the xenografts of each group. (**B**) Tumor inhibition (%) of the xenografts of each group on the 6th weekend of the experiment. *p<0.001, *vs*. control group; **^#^** *p*<0.01, *vs*. TIMP-2 group. (**C**) Kaplan-Meier survival curves for the xenograft mice of each group (log-rank test, *p* = 0.049). **P = 0.022, *vs*. control group. All experiments were performed in triplicate with consistent results.

VM in histology appears as multiple, ECM-rich PAS positive networks and surround clusters of tumor cells, according to Seftor [11]; any structure containing CD31-positive immunoreactivity was defined as a blood vessel, while VM structures were strictly defined as CD31-negative PAS-positive structures. In this experiment, we investigated the inhibitory effect of NCTD on VM rather than on angiogenesis. As shown in Fig.2, in control group, hematoxylin and eosin (H&E) staining showed VM channels formed by tumor cells and erythrocytes at the center of the channels; CD_31_-PAS double staining showed CD31-negative PAS-positive substances lining channels and forming basement membrane-like structures (VM) with single erythrocyte inside (Fig.2A and 2B). Transmission electron microscopy (TEM) clearly visualized several erythrocytes at the central of the tumor nests in control group and non-vascular structure between the surrounding tumor cells and erythrocytes (Fig.2C). Thus, it is identified that VM existed in GBC-SD nude mouse xenografts (9/10, 90.0%). However, microscopically similar phenomenon failed to occur in the xenografts in TIMP-2 or NCTD group, with destroyed cellular organelles, cell necrosis, nuclear pyknosis, fragmentation and apoptotic bodies (Fig.2A∼C). The results shown that highly aggressive GBC-SD cells were able to form VM network structures when injected subcutaneously into the mice, and facilitated growth of GBC-SD xenografts; that NCTD, similar to TIMP-2, inhibited the VM formation of GBC-SD xenografts, and then suppressed tumor growth of the xenografts effectively and safely *in vivo*.

**Figure 2:** Effect of NCTD on VM channels of GBC-SD xenografts *in vivo*. (**A**: H&E staining, **B**: CD_31_-PAS double staining, original magnification, ×400; **C**: TEM, original magnification, ×8000). In control group, H&E staining showed tumor cell-lined VM channels containing red blood cells (***yellow arrow***) without any evidence of tumor necrosis; CD_31_-PAS double staining showed PAS-positive substances lining channels and forming basement membrane-like structures (VM) with single red blood cell inside (***yellow arrows***), and endothelium-dependent vessels (***white arrows***) presenting in the same field with VM; TEM visualized several red blood cells at the central of tumor nests in the xenografts (***red arrow***). However, similar phenomenon failed to occur in the xenografts in TIMP-2 group or NCTD group, with destroyed cellular organelles, cell necrosis (***blue arrows***), nuclear pyknosis, fragmentation and apoptotic bodies (***brown arrows***).

### NCTD inhibits VM-like network formation of GBC-SD cells *in vitro*

To further verify the anti-VM activity of NCTD, in this experiment we observed the vasculogenic-like networks formed from 3-D matrix of GBC-SD cells *in vitro* under an inverted phase-contrast light microscope and an electron microscopy. In control group, GBC-SD cells were able to form hollow tubular network structures and microstructures when cultured on Matrigel and rat-tail collagen type I composed of the ECM gel in the absence of endothelial cells and fibroblasts (Fig.3, Fig.4A and 4B). GBC-SD cell-formed networks initiated formation within 48 hours after seeding the cells onto the matrix, matured basically after one week, with optimal structure formation achieved by two weeks (Fig.3 and Fig.4); and as an ingredient of VM base-membrane, PAS positive, cherry-red materials secreted by GBC-SD cells were found in granules and patches in the cytoplasm of GBC-SD cells appeared around the signal cell or cell clusters by PAS staining without hematoxylin counterstain (Fig.4C). But in the process of network formation, using TIMP-2 or NCTD for 2 days, GBC-SD cells lost the capacity of the above vasculogenic-like network formation, with visible cell aggregation, float, nuclear fragmentation (Fig.3). Furthermore, using TIMP-2 or NCTD for 2∼4 days after network formation, the already formed vasculogenic-like network structures from the 3-D matrix of GBC-SD cells were inhibited or destroyed, with visible cell aggregation, float, deformed collagen framework, decreased microvilli, vacuolar degeneration, nuclear fragmentation and typical apoptotic bodies (Fig.4A∼D). It was showed that the same as TIMP-2, NCTD inhibited and destroyed forming-VM and formed-VM from the 3-D cultures of GBC-SD cells *in vitro*, thus confirmed the anti-VM activity of NCTD for gallbladder cancers *in vitro*.

**Figure 3:** Effect of NCTD on the forming VM-like networks of the 3-D matrix of GBC-SD cells *in vitro*. GBC-SD cell-formed networks in control group initiated formation within 48 hr after seeding the cells onto the matrix, matured basically after 1 week, with optimal structure formation achieved by two weeks; but in the process of network formation, using TIMP-2 or NCTD for 2 days, GBC-SD cells lost the capacity of the above vasculogenic-like network formation, with visible cell aggregation, float, nuclear fragmentation.

**Figure 4:** Effect of NCTD on the formed VM-like networks of the 3-D matrix of GBC-SD cells *in vitro*. GBC-SD cells formed the optimal patterned, vasculogenic- like networks when cultured on Matrigel (**A**) and rat-tail collagen I matrix (**B**) for 2 weeks, PAS positive, cherry-red materials found in granules and patches in the cytoplasm appeared around the signal cell or cell clusters by PAS staining without hematoxylin counterstain (**C**); and channelized or hollowed vasculogenic-like network microstructures visualized under electron microscopy (**D**, TEM ×1200) with clear microvilli surrounding cluster of tumor cells (***red arrow***), cellular organelle structures, and cell connection with an increased electron density in density (***yellow arrow***). After this, using TIMP-2 or NCTD for 2-4 days, the already formed VM-like networks from the 3-D matrix of GBC-SD cells were inhibited or destroyed, with visible deformed collagen framework, decreased microvilli, destroyed cellular organelles, vacuolar degeneration (***green arrow***), nuclear fragmentation (***brown arrows***), and typical apoptotic bodies (***white*** ** ***arrows***).

### NCTD affects malignant phenotypes of GBC-SD cells *in vitro*

To confirm the inhibitory effect of NCTD on VM-like network formation of GBC-SD cells, we further observed effects of NCTD on malignant phenotypes of GBC-SD cells such as proliferation, apoptosis, invasion and migration *in vitro* by tetrazolium-based colorimetric (MTT) assay, flow cytometry (FCM), Matrigel-coated transwell system and collagen gel contraction test. As shown in Fig.5, after NCTD treatment, the morphology of GBC-SD cells showed visible cell aggregation, float, nuclear fragmentation, cataclysm; a significant inhibition of proliferation of GBC-SD cells was showed in a dose-dependent manner with the NCTD IC_50_ value 56.18 µg/ml, as compared to control groups (Fig.5A). These observations were confirmed by apoptotic assay *via* FCM and microstructure observation under TEM which revealed that GBC-SD cell apoptosis were significantly induced in a dose-dependent manner as compared to control group (*p*<0.001), i.e., apoptosis percent of GBC-SD cells (total cells under right quadrant of cells) increased (Fig.5B); and that microvillus decreasing, cytoplast vacuole, nuclear shrinkage, chromatin aggregation and typical apoptosis bodies in NCTD group were observed under TEM (Fig.4D). In addition, the invaded number of GBC-SD cells in NCTD or TIMP-2 group was much less than that of control group (*p*<0.0001; Fig.6A); a significant difference of gel contraction index (CI) of GBC-SD cells was observed between control group and TIMP2 or NCTD group from 1 to 4 days (*p<0.01, *vs*. TIMP2 or NCTD group), without different CI between TIMP-2 group and NCTD group (Fig.6B). The results shown that NCTD inhibited significantly proliferation, invasion and migration of GBC-SD cells, and induced apoptosis of GBC-SD cells *in vitro* in a dose dependent manner as compared to control group. Taken together, these *in vitro* results indicated that NCTD affected these malignant phenotypes of GBC-SD cells, thus inhibited VM-like network formation of GBC-SD cells.

**Figure 5:** Effects of NCTD on proliferation and apoptosis of GBC-SD cells *in vitro*. (**A**) Inhibition of NCTD on proliferation of GBC-SD cells by MTT assay (magnification×400) and the dose-response curves of NCTD effect on GBC-SD cells with the IC_50_ value of 56.18 µg/ml. (**B**) Inducement of NCTD on apoptosis of GBC-SD cells by flow cytometry [in FCM scatter diagram, the left lower quadrant show live cells (FITC-/PI-), the right upper quadrant for necrotic or death cells (FITC+/PI+), and the right lower quadrant for apoptotic cells (FITC+/PI-)]. No apoptotic cells were observed in control group (0 µg/ml of NCTD). After treatment with NCTD for 24 hr and with the concentration increasing, GBC-SD cell apoptosis was increased significantly as compared to control group (*p*<0.001), with a dose- dependent manner. Three separate experiments were performed, with consistent results.

**Figure 6:** Effects of NCTD on invasion and migration of GBC-SD cells *in vitro*. (**A**) Inhibition of NCTD (1/2 IC_50_ dose) on invasion of GBC-SD cells by transwell invasion assay with H&E staining (magnification×200). The invaded number of GBC-SD cells in NCTD or TIMP-2 group was much less than that of control group (*p*<0.0001). (**B**) Inhibition of NCTD (1/2 IC_50_ dose) on migration of GBC-SD cells by collagen gel contraction test. A significant difference of gel contraction index (CI) of GBC-SD cells was observed between control group and TIMP2 or NCTD group from 1 to 4 days (*p<0.01, *vs*. TIMP2 or NCTD group), without different CI between TIMP-2 group and NCTD group. All experiments were performed in triplicate with consistent results.

### NCTD downregulates expression of VM signaling-related markers EphA2, FAK and Paxillin-P of GBC-SD nude mouse xenografts *in vivo*

To investigate the underlying mechanisms of NCTD effects on tumor growth and VM of human gallbladder cancers, in this study we explored the *in vivo* regulation effect of NCTD on the EphA2/FAK/Paxillin signaling pathway, i.e., expression of VM signaling-related markers EphA2, FAK and Paxillin-P at protein and mRNA levels of GBC-SD xenografts by indirect immunofluorescence method, western blotting and RT-PCR. We found that expression (bright yellow-green fluorescent staining reactant in the cytoplasm, or western gray value) of EphA2, FAK and Paxillin-P proteins in NCTD or TIMP-2 group was significantly downregulated when compared with control group (Fig.7A and 7B; all *p<0.001). Expression of EphA2, FAK and Paxillin-P mRNAs in NCTD or TIMP-2 group was also significantly downregulated as compared to control group (Fig.7C; all *p<0.001). No statistical difference on expression of these VM signaling-related markers was observed between NCTD group and TIMP-2 group. We previously reported that highly aggressive GBC-SD cells overexpressed EphA2, FAK and Paxillin-P formed *in vitro and in vivo* VM networks through the activation of the EphA2/FAK/Paxillin signaling pathway; and TIMP-2 effectively inhibited expression of these VM signaling-related markers, i.e., the EphA2/FAK/Paxillin signaling pathway, thus inhibiting VM of GBC-SD cells *in vitro and in vivo* [42]. The results in this study showed that highly aggressive GBC-SD cells formed *in vivo* VM networks by overexpressing EphA2, FAK and Paxillin-P proteins/mRNAs; NCTD downregulated expression of these VM signaling-related markers *in vivo*, thus similarly to TIMP-2, inhibited VM formation of GBC-SD cells and growth of GBC-SD xenografts. These findings demonstrated that NCTD inhibits tumor growth and VM of human gallbladder cancers, probably *via* blocking the EphA2/FAK/Paxillin signaling pathway.

**Figure 7:** Expression of VM signal-related marker EphA2, FAK and Paxillin-P of GBC-CD xenografts *in vivo* (A, indirect immunofluorescence, original magnification, ×400; B, Western blotting; C, RT-PCR). (**A** and **B**): Expression (bright yellow-green fluorescent staining reactant in the cytoplasm, or western gray value) of EphA2, FAK and Paxillin-P proteins of the xenografts in TIMP-2 or NCTD group was significantly down-regulated as compared to control group (*p<0.001), without difference on expression of these proteins between NCTD group and TIMP-2 group. (**C**) Expression of EphA2, FAK and Paxillin-P mRNAs of the xenografts in TIMP-2 or NCTD group was also down-regulated significantly as compared to control group (*p<0.01). No significant difference on expression of these mRNAs was observed between NCTD group and TIMP-2 group.

## Discussion

VM is a newly-defined tumor microcirculation pattern in some highly aggressive malignant tumors, which differs from endothelium-dependent angiogenesis, and is associated with a poor prognosis for the patients with some aggressive malignancies such as melanoma and gallbladder cancers [11], [14]–[18]. Because VM is an alternative pathway for highly aggressive tumors to guarantee their blood supply, whereas not an angiogenic event arising from pre-existing vessels, it is necessary to find potential therapeutic approaches for targeting VM or in addition to antiangiogenic therapies [23]–[25]. We reported that VM existed in human gallbladder cancers, highly aggressive gallbladder cancer GBC-SD cells and xenografts; whereas poorly aggressive SGC-996 cells did not form the VM networks under the same conditions [13], [17], [18], [42]. In this study, the results showed that NCTD, similar to TIMP-2, inhibited tumor growth and VM formation of GBC-SD xenografts, and prolonged survival time of the xenograft mice. These results were confirmed by the fact that inhibition and destruction of forming-VM and formed-VM from the 3-D matrices, and influence of the malignant phenotypes, i.e. proliferation, apoptosis, invasion, migration of GBC-SD cells *in vitro*. Overall, we show evidence that NCTD inhibits tumor VM and prolongs host survival in highly aggressive gallbladder cancers.

The molecular mechanisms underlying VM displayed by highly aggressive malignant tumor cells, especially, highly aggressive gallbladder cancers remain poorly understood. Therefore, understanding the key molecular mechanisms that regulate tumor VM would be an important event and provide potential targets for new cancer therapies. Recently, some experiments have shown the importance of several key molecules or signaling pathways in promoting cell migration, invasion and matrix remodeling, in particular, VM formation by aggressive malignant tumor cells, including phosphoinositide 3-kinase (PI3K), matrix metalloproteinases (MMPs), laminin-5γ2 (Ln-5γ2) chain, epithelial cell kinase (ECK2)/EphA2, FAK, tissue factor and its pathway inhibitor and vascular endothelial growth factor α, and others [12]. We recently reported that VM formation in gallbladder cancers through the activation of a key VM-related signaling pathway—the EphA2/FAK/Paxillin signaling pathway in the 3-D matrices of highly aggressive GBC-SD cells *in vitro* and GBC-SD nude mouse xenografts *in vivo* [42]. The EphA2/FAK/Paxillin signaling pathway is a key pathway which regulated VM formation of aggressive malignant tumor cells. Of them, EphA2, a member of the Eph (ephrin­receptor) family of protein tyrosine kinases which could be pivotal factors of VM and an upstream molecule to regulate VM formation, has been found to play an important role in angiogenesis and in the process of formation of VM [42]–[45]. Knockdown of EphA2 expression does result in a redistribution of EphA2 on the cell membrane, and an inability of cells to form vasculogenic structures. Transient knockout of EphA2 *in vitro* abrogated the ability of highly aggressive melanoma cells to form the vasculogenic-like networks [46], [47]. FAK, a non-receptor protein tyrosine kinase, is an important key mediator of the aggressive melanoma phenotype including VM, through Erk1/2 and unknown downstream effectors to regulate or promote invasion and migration of aggressive melanoma cells that may contribute to an increase of VM potential; moreover, Erk1/2 regulates MMP-2 and membrane type 1-MMP (MT1­MMP) activity, thus promoting melanoma invasion and VM [48], [49]. Paxillin, a focal adhesion-associated phosphotyrosine-containing docking protein, recruit signaling molecules to a specific cellular compartment, the focal adhesions, and/or to recruit specific combinations of signaling molecules into a complex to coordinate downstream signaling and regulate cell spreading and motility [50]. In VM, activity of FAK, as bridging protein between EphA2 and integrins, mediates Paxillin phosphorylation at local adhesion sites, then regulating focal adhesion effect, increasing tumor cell mobility, being conducive to the formation of VM [45]. Therefore, as a key pathway which regulated VM formation of aggressive malignant tumor cells, the EphA2/FAK/Paxillin signaling pathway may represent predominant targets for anti-VM of tumors and cancer therapy.

We previously reported that highly aggressive GBC-SD cells overexpressed EphA2, FAK and Paxillin-P formed VM networks through the activation of the EphA2/FAK/Paxillin signaling pathway [42]. In this study, we found that expression of EphA2, FAK and Paxillin-P at protein and mRNA levels in NCTD group was significantly downregulated (all *p*<0.001), and no statistical difference on expression of these VM signaling-related genes was observed between NCTD group and TIMP-2 group. The results showed that NCTD inhibits tumor VM and prolongs host survival in highly aggressive gallbladder cancers, probably *via* blocking the EphA2/FAK/Paxillin signaling pathway.

Gallbladder cancer is a lethal and aggressive malignant neoplasm. The only potentially curative therapy for this disease is surgical resection. Unfortunately, most patients with gallbladder cancer present with advanced and unresectable disease and only 10%∼30% of the patients are indicated for surgery on presentation or palliative treatment such as chemotherapy and radiotherapy, whereas these adjuvant therapies for the disease are disappointing. In view of the high aggressive and much VM of gallbladder cancer and the multiple antitumor activities of NCTD, in this study we observed if NCTD has the anti-VM activity against highly aggressive gallbladder cancer and the underlying mechanisms in order to serve as a VM inhibitor and an adjuvant therapy for human gallbladder cancer. NCTD, a demethylated derivative of cantharidin with anti-tumor, is used clinically as a routine anticancer drug in China because of its relatively synthesized facility, strong anticancer activity with less side-effect [33]–[38]. However, the exact antitumor mechanisms remain to be not thoroughly elucidated.

Recently, several lines of evidence suggested that NCTD-induced apoptosis in the anticancer effects on human tumor cells, such as leukemia K562 cells, HL-60 cells and GBC-SD cells, might correlate with arresting the cell cycle at G_2_/M phase, inhibiting DNA synthesis, influencing cell metabolism, regulating apoptotic-related genes through mitochondrial and caspase pathways, and mitogen-activated protein kinases (MAPKs), including extracellular signal-regulated kinase (ERK), c-Jun-NH_2_- terminal kinase (JNK) and p38^MAPK^ [36]-[40], [51]-[60]. Lately, there is a growing interest that some anticancer researches for NCTD have begun to focus on antiangiogenesis and anti-VM. We firstly reported the *in vitro* and *in vivo* antiangiogenic activity of NCTD as a potential angiogenic inhibitor for gallbladder cancers [41], [61]. Chen et al also reported the *in vitro* and *in vivo* antiangiogenic effect of NCTD on CT26 cells by down-regulation of MAPK expression of phosphorylated (p)-JNK and p-ERK, and considered NCTD is a synthetic, small-molecule compound possessing antiangiogenic activity [62]. In this study, we firstly demonstrated that NCTD inhibits tumor VM and prolongs host survival in highly aggressive gallbladder cancers probably *via* blocking the EphA2/FAK/Paxillin signaling pathway, and could serve as a potential anti-VM agent for human highly aggressive gallbladder cancers. Thus, the results advance our present knowledge concerning the anticancer activities of NCTD and provide the basis for new therapeutic intervention. We believe that NCTD is an effective “more targets” anticancer agent for human gallbladder cancers by “multifactor” and “multi-points priming” mechanisms [51]; that inhibition of gallbladder cancer VM by NCTD *via* blocking the EphA2/FAK/Paxillin pathway may be one of “more targets” anticancer mechanisms of NCTD. It is possible that NCTD may be more effective if used in combination of other anticancer drugs, as McNamara MG et al [63] have suggested, that the future therapeutic spectrum for GBC will likely encompass novel combinations of targeted therapies with cytostatics in scientifically and molecularly directed schedules, thus permitting fewer mechanisms of escape for tumor cells.

## Methods

### Cell culture

Human gallbladder cancer cell lines used in this study were GBC-SD (Shanghai Cell Biology Research Institute of Chinese Academy of Sciences, CAS), which was confirmed to have highly aggressive characteristic [13]. Cells were maintained and propagated in Dulbecco's modified Eagle's media (DMEM, Gibco, USA) supplemented with 10% fetal bovine serum (FBS, Hangzhou Sijiqing Bioproducts, China) and 10^5^ U·ml^−1^ penicillin and streptomycin (Shanghai Pharmaceutical Works, China) in an incubator (Forma series II HEPA Class 100, Thermo, USA) at 37°C with 5% CO_2_.

### Tumor xenograft assay and survival analysis *in vivo*

This study was carried out according to the official recommendations of Chinese Community Guidelines and the ARRIVE (Animal Research: Reporting of *In Vivo* Experiments) guidelines [64]. The protocol was approved by the Committee on the Ethics of Animal Experiments of Tongji Hospital, Tongji University School of Medicine, and the Science and Technology Commission of Shanghai Municipality (Permit Number: SYXK 2012–0031).

Balb/c nu/nu mice (equal numbers of male and female mice, 4-week old, about 20 grams) used in this study were provided by Shanghai Laboratory Animal Center, Chinese Academy of Sciences and housed in specific pathogen free condition. A volume of 0.2 ml serum-free medium containing single-cell suspensions of GBC-SD (7.5×10^6^ ml^−1^) were respectively injected subcutaneously into the right-rear axils of nu/nu mice. The mice, by 2 weeks when a tumor xenograft was apparent in all mice right-rear axils, were randomly divided into a control group (*n* = 10) receiving intraperitoneal (i.p.) injections of 0.1 ml normal saline alone twice each week, a NCTD (Injection solution: 5 mg·ml^−1^; Jiangsu Kangxi Pharmaceutical Works, China; *n* = 10, each mouse receiving i.p. injections of 28 mg/kg NCTD given in 0.1 ml of normal saline) group, and a TIMP-2 recombinant protein (Sigma, Germany; *n* = 10, each mouse receiving intratumoral injection of 5 mg/kg) group, twice each week for 6 weeks in all. The xenograft size i.e. the maximum diameter (a) and minimum diameter (b) were measured with calipers two times each week. The tumor volume was calculated by the following formula: V (cm^3^) = 1/6π*ab* ^2^. Tumor growth curve and tumor inhibitory rate of each group were respectively evaluated. Tumor inhibitory rate  =  (volume in control group - volume in experimental group)/volume in control group×100%. The dose of NCTN in the *in vivo* experiment is 28 mg/kg, i.e., a safe dose of NCTD 1/5 LD_50_ [41]. Survival time of each group was also evaluated. The outcome was followed from the date of NCTD injection to the date of death. The median follow-up period for mice was 15 (range 3–31) weeks. Experiments were performed in duplicate and repeated three times with consistent results.

### VM formation assay of GBC-SD nude mouse xenografts *in vivo*

VM formation assay from xenograft sections of each group *in vivo* was conducted by H&E staining, immunohistochemical CD_31_-PAS double staining and TEM. For H&E staining: paraffin-embedded tissue specimens from the xenograft were deparaffinized, hydrated, and stained with H&E. Companion serial section were stained with double staining of CD_31_ and PAS: sections from paraffin-embedded tissue specimens (4 µm) of the xenografts were deparaffinized, hydrated, and pretreated, they were incubated in turn with mouse monoclonal anti-CD_31_ protein IgG (Neomarkers, USA, dilution: 1∶50), goat anti-mouse Envision Kit (Genetech, USA), 3,3-diaminobenzidine (DAB) chromogen, 0.5% periodic acid solution, followed by treating with Schiff solution in a dark chamber, finally all of these sections were counterstained with hematoxylin, observed under a light microscope (Olympus IX70, Japan). For TEM, fresh xenograft tissue samples (0.5 mm^3^) of each group were fixed in cold 2.5% glutaraldehyde in 0.1 mol^.^L^−1^ of sodium cacodylate buffer and postfixed in a solution of 1% osmium tetroxide, dehydrated, and embedded in a standard fashion. The specimens were then embedded, sectioned, and stained by routine means for a JEOL-1230 TEM (Japanese Electronics, Japan). All experiments were performed in triplicate.

### Vasculogenic-like network assay of 3-D matrix of GBC-SD cells *in vitro*

Matrigel and rat-tail type I collagen 3-D matrices were prepared as described previously [13]. Cells were allowed to adhere to matrix, and untreated (control group) and treated with 100 nM TIMP-2 recombinant protein (Sigma, Germany; TIMP_2_ group) or 28 µg·ml^−1^ of NCTD (a dose of NCTD 1/2 IC_50_, NCTD group) for 2 days. The ability of GBC-SD cells to engage in VM was respectively analyzed using immunohistochemistry and TEM. Immunocytochemistry included H&E staining and PAS staining (without hematoxylin counterstain). The outcome was observed under a light microscope with×10 and ×40 objectives. The images were taken digitally using a Zeiss Televal invertal microscopy (Carl Zeiss, Inc., Thornwood, NY) and camera (Nickon, Japan) at the time indicated. Also, the 3-D culture specimens were fixed, post-fixed, dehydrated, embedded, sectioned, and stained by above routine means for a JEOL-1230 TEM. All experiments were also performed in triplicate.

### Analyses of malignant phenotypes including proliferation, apoptosis, invasion and migration of GBC-SD cells *in vitro*

The cultured GBC-SD cell suspensions were used for proliferation assay *via* MTT method and apoptosis assay *via* FCM *in vitro*. Cells were cultured in a 96-well plate (3×10^5^ cells/ml·100 µl/well) in culture medium overnight, then treated with various concentrations of NCTD in fresh culture medium at 37°C in 5% CO_2_ for 24 hours. MTT (Sigma, MO, USA) assay was used to determine the effect of NCTD on proliferation of GBC-SD cells. The optical densities (*A* value) at 540 nm were measured with an enzyme-linked immunosorbent assay reader (Biorad model 450, Sigma, Germany). The *A*540 value of the experimental groups was divided by the *A*540 value of untreated controls and presented as a percentage of the cells. The inhibitory percent of NCTD on GBC-SD cells (%)  =  (1-*A*540 value in the experimental group /*A*540 value of control group) ×100%. Three separate experiments were performed. The concentration of drug giving 50% growth inhibition (IC_50_) was calculated from the formula IC_50_ = lg^-1^[Xm-I (p-0.5)].

For FCM, cells (3×10^5^ cells/ml·100 µl/well) cultured in a 96-well plate in culture medium were untreated (negative control) or treated with various concentrations (5.0∼50.0 µg/ml, experimental groups; 6 wells per concentration) of NCTD at 37°C in 5% CO_2_ for 24 hours, then were made up into the cell suspension (5×10^5^ cells/ml), and suspended in 500 µl Binding Buffer. Tumor DNA was then stained for 15 minutes with 5 µl Annexin V-FITL and propidium iodine (PI, Sigma, USA). DNA value and apoptotic rate of each group were determined by Cell Apoptotic Detection Kit (BioDev, China) and Fluorescent Activated Cell Sorter (420 type FACS Flow cytometry, Becton-Dickinson, CA). Three separate experiments were performed.

The 35-mm, 6-well Transwell membranes (Coster, USA) were used to measure the *in vitro* invasiveness, i.e., invasion assay of GBC-SD cells. Briefly, a polyester membrane with 8-µm pores was uniformity coated with a defined basement membrane matrix consisting of 50 µl Matrigel (Becton Dickinson, USA) mixture which diluted with serum-free DMEM (2 volumes *versus* 1 volume) over night at 4°C and used as the intervening barrier to invasion. Upper wells of chamber were respectively filled with 1 ml serum-free DMEM containing 2×10^5^ ml^−1^ GBC-SD cells (n = 3). Cells were respectively untreated (control group) and treated with recombinant TIMP-2 (≤100 nM, Sigma, Germany; TIMP_2_ group) or 28 µg·ml^−1^ of NCTD (a dose of NCTD 1/2 IC_50_, NCTD group) in fresh culture medium (0.3 ml/every chamber) for 24 hour. Lower wells of chamber were filled with 3 ml serum-free DMEM containing 1×MITO+ (Collaborative Biomedical, Bedford, MA). After 24 hour in a humidified incubator at 37°C with 5% CO_2_, cells that had invaded through the basement membrane were stained with H&E, and counted under a light microscopy. Invasiveness was calculated as the number of cells that had successfully invaded through the matrix-coated membrane to the lower wells. Briefly, quantification was done by counting the number of cells in 5 independent microscopic fields at a 400-fold magnification. Experiments were performed in duplicate and repeated three times with consistent results.

Collagen gel suspensions for GBC-SD cell lines are prepared by mixing 250 µl of a suspension that contained 3×10^6^ ml^−1^ into 250 µl of undiluted rat-tail collagen type I (Sigma, Germany; 4.25 mg^.^ml^−1^) dripped into sterilized 35-mm petridishes that contained 2 ml culture medium to prevent adhesion of the collagen to the glass substrate. The suspensions are allowed to polymerize for 1 hour at room temperature before these culture dishes were placed in the 37°C with 5% CO_2_ incubator. Cells were treated according to above invasion assay. Gel contraction was defined as the relative change in the gel size, measured in two dimensions, including maximum and minimum diameters. The gel measurements were recorded daily, and the culture medium was changed every one day. Contraction index (CI) was calculated i.e., migration assay, as follows: CI = 1-(D-D_0_)^2^×100%, where D is the primary diameter of rat-tail collagen type I, D_0_ is the average of maximum and minimum diameters of gel. All experiments were performed in triplicate.

### Detections of VM signaling-related markers EphA2, FAK and Paxillin-P using immunofluorescence, western blotting and RT-PCR

Expression of EphA2, FAK and Paxillin-P proteins from the GBC-SD nude mouse xenografts of each group were respectively determined by indirect immunofluorescence method and western blotting. For immunofluorescence detection, the frozen sections (4 µm) of the xenografts from each group were pretreated with 99.5% acetone, methanol with 3% hydrogen peroxide and 20% normal goat serum, were added in order with 50 µl (1∶100) primary antibody [rabbit anti-human polyclonal antibody; EphA2 and FAK, Santa Cruz, USA; Paxillin (phosphor Y118), Abcam, USA], biotinylated secondary antibody (1∶100; goat anti-rabbit IgG-FITC/GGHL-15F, Immunology Consultants Laboratory, USA), respectively. Then, sections were rinsed in TBS solution and distilled water, mounted coverslip using buffer glycerine, and observed under a fluorescence microscope (Nikon, Japan). For negative control, the slides were treated with PBS in place of primary antibody. Ten sample slides in each group were chosen by analysis. More than 10 visual fields were observed per slide. Expression of each protein on slides of the xenografts showed a yellow-green fluorescent dyeing. The fluorescent dyeing intensity was classed into -, ±, +, ++, +++, ++++. Of them, -∼+: negative expression, ≥++: positive expression. For western blotting, cells were lysed with 200 µl of cell lysis buffer (protein extraction kit, KangChen, KC-415, China) containing a cocktail of protease inhibitors and the supernatant of the lysed cells was recovered. BCA protein quantitative determination was carried out with a protein quantitative kit (KangChen, KC-415). Then, an aliquot of 20 µg of proteins was subjected to sodium dodecyl sulfate- polyacrylamide gel electrophoresis (SDS-PAGE) for electrophoresis under reducing condition, and were then transferred to a PVDF membrane. An hour after being blocked with PBS containing 5% non-fat milk, the membrane was incubated overnight, was then added in order with each primary antibody [(mouse anti-human antibody, 1∶3000; EphA2, FAK: Santa Cruz; Paxillin (phosphor Y118): Abcam)], and mouse anti-human GAPDH antibody (1∶10000; Kangcheng Bioengineering, Shanghai) diluted with PBST containing 5% non-fat milk at 4°C, an appropriate anti-mouse HRP-labeled secondary antibody (1∶5000; Kangcheng Bioengineering). The target proteins were visualized by an enhanced chemiluminescent (ECL) reagent (KC chemiluminescent kit, KangChen, KC-420), imaged on the Bio-Rad chemiluminescence imager. The gray value and gray coefficient ratio of every protein were analyzed and calculated with Image J analysis software.

Expression of EphA2, FAK and Paxillin-P mRNAs from the xenografts of each group were determined by semi-quantitative RT-PCR assay. RT-PCR was performed as described by the manufacturer. Total RNA was extracted from the xenograft cells using the Trizol reagent (Invitrogen, USA). Concentration of RNA was determined by the absorption at 260∼280. The primers for amplification were designed and synthesized by Shanghai Kangcheng Bioengineering. The primers for EphA2, FAK, Paxillin-P and GAPDH were as follows: EphA2 (140 bp) 5'TTA GGG AGA AGG ATG GTG AGT T 3' (sense), 5'GTT GCT GTT GAC GAG GAT GTT3' (anti-sense); FAK (152 bp) 5'CCC AGA AAG AAG GTG AAC G3' (sense), 5'GGT CGA GGG CAT GGT GTA3' (anti-sense); Paxillin-P (228 bp) 5'CTT CAA GGA GCA GAA CGA CAA A3' (sense), 5'TAG CAG GTG GTA GGG ACG AGA3' (anti-sense); GAPDH (211 bp) 5'CCT CTA TGC CAA CAC AGT GC3' (sense), 5′GTA CTC CTG CTT GCT GAT CC3′ (anti-sense). PCR was performed in a 20 µL reaction volume. RT-PCR reaction was run in the following condition: GAPDH, at 95°C for 5 minutes; at 95°C for 10 seconds, at 57°C for 15 seconds, at 72°C for 20 seconds, at 85.5°C (fluorescence collection) for 5 seconds, 35 cycles; at 72∼99°C for 5 minutes. EphA2, at 95°C for 5 minutes; at 95°C for 10 seconds, at 60°C for 15 seconds, at 72°C for 20 seconds, at 84°C (fluorescence collection) for 5 seconds, 35; at 72∼99°C for 5 minutes. FAK, at 95°C for 5 minutes; at 95°C for 10 seconds, at 60 °C for 15 seconds, at 72°C for 20 seconds, at 82.3°C (fluorescence collection) for 5 seconds, 35; at 72∼99°C for 5 minutes. Paxillin-P, at 95°C for 5 minutes; at 95°C for 10 seconds, at 60°C for 15 seconds, at 72°C for 20 seconds, at 86°C (fluorescence collection) for 5 seconds, 35; at 72∼99°C for 5 minutes. 10 µL PCR products was placed onto 15 g/L agarose gel and observed by EB (Ethidium Bromide, Huamei Bioengineering, China) staining using the ABI Prism 7300 SDS Software.

### Statistical analysis

All data were expressed as mean ± SD and performed using SAS version 9.0 software (SAS Institute Inc., USA). Statistical analyses to determine significance were tested with the *χ* ^2^, *F* or Student-Newman-Keuls *t* tests. Log-rank test and Kaplan-Meier survival curves were constructed for the selected variables. *p*<0.05 was considered statistically significant.
